# Intravascular NK-cell lymphoma: a case report and review of the literature

**DOI:** 10.1186/s13000-015-0336-7

**Published:** 2015-07-01

**Authors:** Yalan Bi, Zhen Huo, Zhiyong liang, Yunxiao Meng, Congwei Jia, Xiaohua Shi, Lan Song, Yufeng Luo, Qing Ling, Tonghua Liu

**Affiliations:** Department of Pathology, Peking Union Medical College Hospital, Chinese Academy of Medical Sciences and Peking Union Medical College, No.1 Shuaifuyuan, Wangfujing, DongCheng District, Beijing, 100730 China; Department of Radiology, Peking Union Medical College Hospital, Chinese Academy of Medical Sciences and Peking Union Medical College, Beijing, China

**Keywords:** Intravascular lymphoma, NK-cell lymphoma, Epstein-Barr virus

## Abstract

**Background:**

Intravascular NK-cell lymphoma (IVNKL) is an extremely rare variant of non-Hodgkin lymphoma. To our knowledge, there are only a few cases reported in the English literature. Here, a case of a 29-year-old male with IVNKL involving the skin of the trunk and 4 extremities and liver is presented. A comprehensive literature review is undertaken to summarize the clinical and pathological features of this disorder.

**Findings:**

In our case, large neoplastic lymphoid cells are restricted to the lumen of small vessels and exhibit the phenotype of a true NK cell. The morphology and immunophenotype, positivity of EBER and NK-cell origin are similar to other IVNKL cases. In addition, some cases including ours carry a poor prognosis as multiple systems or vital organs are involved.

**Conclusion:**

In summary, we report a case of an unusual intravascular lymphoma of NK-cell lineage that displays both clinical and pathological features and compare it with other differential diagnoses. It is important to recognize this rare entity to make an appropriate diagnosis and achieve a better understanding regarding the treatment and prognosis.

## Background

Intravascular NK-cell lymphoma (IVNKL) was first reported by Santucci et al. in 2003 [1] and is revealed as an infiltration of large cells with an NK/T-cell phenotype (CD3ε+, CD56+, and markers for cytotoxicity +) that is localized strictly intravascularly. Most of these cases are Epstein-Barr virus nucleic acid EBER (Epstein-Barr virus-encoded small RNA) positive and T-cell receptor (TCR) gene rearrangement negative. Multiple organs may be involved, resulting in a variety of clinical presentations; however, the most common locations that are involved are the skin and the central nervous system (CNS). IVNKL is an aggressive lymphoma with a variable but mostly limited response to chemotherapy and an overall poor prognosis, especially for those patients with multi-system involvement.

Intravascular lymphoma (IVL) is a rare entity. This disorder was first described as angioendotheliomatosis proliferans systemisata by Pfleger and Tappeiner [2] in 1959. The neoplastic cells were initially believed to be of endothelial origin; however, subsequent immunohistochemical and molecular studies demonstrated the lymphoid nature of the neoplastic cells [3]. Most cases constitute a variant of an extranodal diffuse large B-cell lymphoma, and only approximately 10 % of the published cases are of T-cell or histiocytic origin [4]. To date, relatively few cases with an NK-cell lineage have been reported in the English literature (Table 1) [1, 5–12].

**Table 1:** Characters of reported cases of IVNKL

Case number/case	Age/gender	Involved organ(s)	Treatment and follow up							
1. Santucci et al. [1]	54/M	Skin, CNS	Chemotherapy, died 17 months after diagnosis							
2. Wu et al. [5]	41/M	Skin	Chemotherapy, alive and event free at 12 months							
3. Wu et al. [5]	47/F	CNS, bone marrow, kidneys, ovaries, cervix	Treatment unclear, died half a month after diagnosis							
4. Kuo et al.[6]	71/F	Skin	Alive 5 months after diagnosis without treatment							
5. Song et al. [7]	40/F	Skin	Chemotherapy, alive and event free at 7 months							
6. Nakamichi et al.[8]	23/F	Skin	Chemotherapy and stem cell transplantation, died of acute GVHD 9 months after diagnosis							
7. Cerroni et al. [9]	63/M	Skin	Chemotherapy, died 6 months after diagnosis							
8. Liao et al. [10]	42/F	Skin	Chemotherapy and radiotherapy, alive with disease 14 months after diagnosis							
9. Gebauer et al.[11]	72/M	Skin, bone marrow, CNS	Chemotherapy, died 7 months after diagnosis							
10. Liu et al. [12]	37/F	Skin, CNS	Chemotherapy, died 13 months after diagnosis							
11.our case	29/M	Skin, liver	Chemotherapy, died 3 months after diagnosis							
Case number/case	Immunophenotypes									PCR-TCR
	CD3	CD4	CD5	CD8	CD20	CD30	CD56	Cytotoxic markers	EBER	
1. Santucci et al. [1]	+	-	NA	-	-	+	+	+	+	ND
2. Wu et al. [5]	+	-	-	-	-	-	+	+	+	P
3. Wu et al. [5]	+	-	-	-	-	NA	+	+	-	P
4. Kuo et al. [6]	+	-	-	-	-	-	+	+	+	P
5. Song et al. [7]	+	-	NA	-	-	NA	+	+	+	P
6. Nakamichi et al.[8]	+	NA	NA	NA	-	NA	+	+	+	ND
7. Cerroni et al. [9]	+	-	NA	-	-	NA	+	+	+	P
8. Liao et al.[10]	+	-	-	-	-	-	+	+	+	ND
9. Gebauer et al.[11]	+	-	NA	-	-	-	+	+	+	P
10. Liu et al. [12]	+	-	-	-	-	-	+	+	+	ND
11.our case	+	-	-	-	-	+	+	+	+	P

*M*, male; *F*, female

*GVHD*, graft-versus-host disease

*NA*, not available

cytotoxic markers, TIA-1 and/or granzyme B and/or perforin

*PCR-TCR*, polymerase chain reaction analysis of the T-cell receptor g gene

*P*, polyclonal smear

Here, we report on a 29-year-old male patient with IVNKL of the skin with secondary involvement of the liver and provide a brief literature review, aiming to (i) emphasize the diagnostic histopathologic features of this disease, (ii) avoid the trap of misdiagnosis of malignant or benign diseases, and (iii) achieve a better understanding of the character and treatment of this disease.

## Findings

A 29-year-old man presented with erythematous plaques on the thighs and trunk, low fever, intermittent headaches, weight loss and leukopenia. His family history was significant, as his only sister had acute myeloid leukemia (M3) several years previously and was cured by chemotherapy. Physical examination revealed painful, subtle, ill-defined, irregular, blanching erythematous patches on the lower and upper extremities and trunk (Fig. 1a and b) and slight hepatosplenomegaly.

**Fig. 1:** **a** and **b** Red-violaceous ill-defined and irregular plaques on the lower extremities and trunk

A biopsy of the erythematous plaques on the right thigh was performed. The specimen consisted of skin and subcutaneous tissue and measured 1.2 × 0.9 × 0.5 cm. The sample was fixed in 10 % buffered formalin and embedded in paraffin. Four-micron sections were cut and stained with hematoxylin and eosin. The cutaneous lesions contained clusters of atypical lymphoid intravascular cells that were occluding and expanding the lumina of the dilated vessels throughout the subcutaneous tissue (Fig. 2a and b). Reactive lymphocytes were observed and were aggregated around the vessels. The tumor cells were discohensive, large, and pleomorphic and had irregular enlarged nuclei with scanty cytoplasms. Mitotic figures and tumor cell necrosis were obvious.

**Fig. 2:** **a** and **b** Intravascular large pleomorphic tumor cells with irregular nuclei and scanty cytoplasm (hematoxylin and eosin stain ×10 and ×100)

Based on immunohistochemical staining, the phenotype of the tumor cells was CD3+, CD43+, CD56+, TIA-1+, CD30+, CD4-, CD5-, CD7-, CD8-, CD20- and CD79a-. Approximately 90 % of the tumor cell nuclei were Ki-67 positive. The vascular endothelial cells were positive for CD31 and CD34, which demonstrated the intravascular nature of the neoplastic cells (Fig. 3a, b, c and d). In situ hybridization for EBER revealed positive signals in virtually all tumor cell nuclei (Fig. 4). DNA extracted from formalin-fixed paraffin-embedded samples was analyzed by polymerase chain reaction (PCR). The molecular study demonstrated a germline configuration of TCR genes without rearrangements (Fig. 5).

**Fig. 3:** **a**, **b** and **c**, Immunohistochemical staining for CD3, CD56 and TIA-1, respectively, showing positive staining in the tumor cells (×100). **d** Blood vessel endothelial cells surrounding the tumor cells identified by positive staining of CD34 (×40)

**Fig. 4:** In situ hybridization for EBER showing strong signals in the tumor cells (×100)

**Fig. 5:** Molecular studies revealed a germline configuration for the T-cell receptor that is consistent with the possibility of an NK-cell origin. (L = Control Size Ladder for samples of unknown quantity and quality, M = DNA ladder marker, TB (A,B,C), TD and TG (A,B) represent 6 tubes of master mixes for targeting different regions of TCR genes)

Further hematologic analysis demonstrated a normal peripheral blood count (White blood cell count, 5.66x10^9^/L, Red blood cell count, 4.20×10^12^/L, Platelet count, 205×10^9^/L) and a deterioration of liver function. A bone marrow biopsy and cytological examination of cerebrospinal fluid revealed no evidence of tumor involvement.

A diagnosis of IVL of the natural killer cell type was established 6 months after the appearance of initial skin lesions. The patient received 2 cycles of combination chemotherapy (cyclophosphamide, Vincristine, Doxorubicin, Dexamethasone; Hyper CVAD). However, clinical and computed tomography scans revealed multiple low-density hepatic masses, indicating liver involvement (Fig. 6a and b). The status of the patient deteriorated rapidly and he had a fever of 38.5°-39 °C. He died of multi-organ failure 3 months after diagnosis.

**Fig. 6:** Pre-contrast CT images showing multiple low-density hepatic masses with hepatosplenomegaly and bilateral pleural effusion (**a**). Post-contrast CT images showing contrast enhancement in the portal venous phase (**b**)

## Discussion

Among the 11 reported cases of IVNKL, including the cases originally published in English and ours, six (54.5 %) were reported from Asia (2 from China, 2 from Taiwan, 1 from Japan and 1 from Korea), which is consistent with the distribution characteristics of extranodal NK/T-cell lymphoma, nasal type, which has a higher incidence in East Asia and Latin America, with EBV infection occurring in some cases [13]. Of the 11 patients, six were female and five were male. The ages ranged from 23 to 72 years (median, 47 years). Dermatological manifestations were observed in 10 (91 %) cases. Multisystem involvement occurred in 5 patients, and 4 of 5 were CNS involvement. After a follow-up that ranged from half a month to 17 months, 7 of 11 patients died, and only 4 of 11 experienced temporary remission.

In the 11 cases in which the morphology of the IVNKL was described, the tumor cells were all confined within the vessels and had large cell sizes with pale or eosinophilic cytoplasms and irregular hyperchromatic nuclei. Mitotic figures and necrosis were routinely observed. In all 11 cases, typical NK cell immunophenotypes were observed: CD3+; CD56+; TIA-1+; granzyme B+; perforin+; CD4-; CD5-; CD8- and CD20-. EBER detection was performed in 11 cases and was positive in 10 of the 11 cases, indicating Epstein-Barr virus (EBV) infection. T-cell gene rearrangement analysis was performed in 7 of the 11 cases and was negative, confirming an NK-cell origin.

For diagnosis, large neoplastic lymphoid cells of IVNKL are restricted to the lumen of small vessels and exhibit the phenotype of a true NK cell, characterized by tumor cells with a CD2+, cytoplasmic CD3ε + and CD56+ immunophenotype and germline configuration of the TCR gene [14]. Tumor cells also expressed cytotoxic granules, including TIA-1, granzyme B and perforin, and were often EBV positive. Thus, the similar morphology and immunophenotype of other cases, positivity of EBER and NK-cell origin help to confirm the diagnosis of our case as IVNKL.

As so far, IVNKL is not classified within the World Health Organization classification subtypes [15]. However, in view of the unique characteristics of this disease, the diagnosis should be independent to collect more data to help with further study of this disease. Because of the similar morphology and immunophenotypes, TCR rearrangement results, and EBV infection status of intravascular NK-cell lymphoma, extranodal NK/T-cell lymphoma, nasal type (ENKTCL) and aggressive NK-cell leukemia [16, 17], we suggest that IVNKL should be distinguished from the other two subtypes. Patients with IVNKL had no nasal symptoms and obvious abnormalities in the peripheral blood but had the hallmark of intravascular dissemination of tumor cells. In ENKTCL and aggressive NK-cell leukemia, tumor cells were distributed in tissues rather than deposited in blood vessels. The other differential diagnoses of IVNKL include IVL of other lineages (in which the tumor cells have typical immunophenotypes, such as being positive for B or T-cell markers), metastatic neoplasms (for example melanoma or breast cancer, which are validated by medical history and immunochemical staining), and numerous inflammatory processes, including drug reactions and insect bites, showing atypical intravascular CD30+ T-cell proliferation mimicking intravascular lymphoma (which includes variable numbers of intravascular CD30-positive cells, but the extent of the intravascular proliferation is much less florid, and the cells show a mixture of CD4 and CD8 positivity without a monoclonal T-cell population by molecular testing) [18].

Regarding etiological hypotheses, we believe that not only EBV infection but also genetic inheritance is somehow involved in the pathogenesis of this rare lymphoma because of this patient’s remarkable family history. IVNKL treatments are ineffective and include chemotherapy, radiotherapy, and even stem cell transplantation, which cannot change the poor prognosis. Because patients with clinical presentation confined to skin have a better prognosis, the poor outcome may be due to multisystem or vital organ involvement.

## Consent

Written informed consent was obtained from the patient’s parents prior to publication of this case report and the accompanying images. A copy of the written consent is available for review by the Editor-in-Chief of this journal.

## Abbreviations

IVNKL: Intravascular NK-cell lymphoma
EBER: Epstein-Barr virus-encoded small RNA
TCR: T-cell receptor
CNS: Central nervous system
IVL: Intravascular lymphoma
DNA: Deoxyribonucleic acid
PCR: Polymerase chain reaction
EBV: Epstein-Barr virus
